# Plasma Small Extracellular Vesicle-Carried miRNA-501-5p Promotes Vascular Smooth Muscle Cell Phenotypic Modulation-Mediated In-Stent Restenosis

This article has been retracted.

**DOI:** 10.1155/2021/6644970

**Published:** 2021-04-21

**Authors:** Xiao-Fei Gao, Zhi-Mei Wang, Ai-Qun Chen, Feng Wang, Shuai Luo, Yue Gu, Xiang-Quan Kong, Guang-Feng Zuo, Xiao-Min Jiang, Guan-Wen Ding, Yan Chen, Zhen Ge, Jun-Jie Zhang, Shao-Liang Chen

**Affiliations:** ^1^Department of Cardiology, Nanjing First Hospital, Nanjing Medical University, Nanjing, China; ^2^Department of Cardiology, Nanjing Heart Centre, Nanjing, China; ^3^Nanjing Foreign Language School, Nanjing, China; ^4^Department of Neurology, Affiliated Drum Tower Hospital of Nanjing University, Medical School, Nanjing, China

## Abstract

Vascular smooth muscle cell (VSMC) phenotypic modulation plays an important role in the occurrence and development of in-stent restenosis (ISR), the underlying mechanism of which remains a key issue needing to be urgently addressed. This study is designed to investigate the role of plasma small extracellular vesicles (sEV) in VSMC phenotypic modulation. sEV were isolated from the plasma of patients with ISR (ISR-sEV) or not (Ctl-sEV) 1 year after coronary stent implantation using differential ultracentrifugation. Plasma sEV in ISR patients are elevated markedly and decrease the expression of VSMC contractile markers *α*-SMA and calponin and increase VSMC proliferation. miRNA sequencing and qRT-PCR validation identified that miRNA-501-5p was the highest expressed miRNA in the plasma ISR-sEV compared with Ctl-sEV. Then, we found that sEV-carried miRNA-501-5p level was significantly higher in ISR patients, and the level of plasma sEV-carried miRNA-501-5p linearly correlated with the degree of restenosis (*R*^2^ = 0.62). Moreover, miRNA-501-5p inhibition significantly increased the expression of VSMC contractile markers *α*-SMA and calponin and suppressed VSMC proliferation and migration; in vivo inhibition of miRNA-501-5p could also blunt carotid artery balloon injury induced VSMC phenotypic modulation in rats. Mechanically, miRNA-501-5p promoted plasma sEV-induced VSMC proliferation by targeting Smad3. Notably, endothelial cells might be the major origins of miRNA-501-5p. Collectively, these findings showed that plasma sEV-carried miRNA-501-5p promotes VSMC phenotypic modulation-mediated ISR through targeting Smad3.

## 1. Introduction

Percutaneous coronary intervention with stent implantation has been an extremely important treatment for patients with coronary artery disease, but it is also blamed for 5%-10% risk of in-stent restenosis (ISR) [1–3], despite drug-eluting stents (DES) are widely used nowadays. The currently accepted causes of ISR are excessive vascular smooth muscle cells (VSMC) hyperplasia and extracellular matrix (ECM) deposition. Responding to vessel injury and local environmental alternations after stent implantation, contractile (also called mature or differentiated) VSMC for hemodynamic regulation can be switched to a synthetic/dedifferentiated phenotype to increase proliferation, migration, and ECM synthesis for tissue reparation or abnormal vessel narrowing [4, 5]. This process of VSMC phenotypic modulation has been studied for decades, but we still do not fully understand the mechanisms well enough to be able to prevent or treat ISR successfully.

miRNAs, a class of short single-stranded RNAs, have been demonstrated to play an important role in VSMC phenotypic modulation, such as miR-143/145 cluster [6] and miR-22 [7] driving VSMC towards the contractile phenotype. Other miRNAs, such as miR-21 [8] and miR-221/222 [9], could drive VSMC towards the synthetic phenotype. Notably, these miRNAs are mainly transported to target cells through small extracellular vesicles (sEV), which can protect the internal miRNAs from being degraded in the circulation and participate in cell-to-cell communication [10–12]. However, there is still a lack of definitive evidence regarding the effects of circulating sEV-carried miRNA in ISR patients. Accordingly, the present study is designed to address the functional effects and underlying mechanisms of plasma sEV-carried miRNA in VSMC phenotypic modulation-mediated ISR.

## 2. Methods

### 2.1. Experimental Animals

Male Sprague-Dawley rats (8 weeks) were obtained from Animal Core Facility of Nanjing Medical University (Nanjing, China). All animal protocols and procedures were performed according to the Guide for the Care and Use of Laboratory Animal published by the US National Institutes of Health (2011) and approved by the Experimental Animal Care and Use Committee of Nanjing Medical University. Rats were housed in a temperature-controlled room with a 12 h light/dark cycle and free access to water and food.

### 2.2. Rat Carotid Artery Balloon Injury Model

The method of rat carotid artery balloon injury (CABI) model has been reported previously [13]. Briefly, 8-week rats were anesthetized with pentobarbital sodium (60 mg/kg, i.p.) and subjected to insertion of Fogarty balloon catheter (2F, Edwards Lifesciences) into the right external carotid artery between the common carotid artery bifurcation and the distal ligation site. In the sham group, the right carotid artery was exposed but not subjected to the insertion of Fogarty balloon. At 28 days after procedure, the rats were sacrificed with an overdose of pentobarbital sodium (200 mg/kg, iv), and their venous blood and carotid arteries were subsequently collected for further study.

### 2.3. Patients

The method and results of ULTIMATE trial have been reported previously [14, 15]. This trial was performed in accordance with Declaration of Helsinki and International conference, and the protocol was approved by the ethics committee of each participating center. All participants have signed written informed consent. Two groups of subjects from ULTIMATE trial were enrolled in this study, including 20 patients with ISR and 20 patients without ISR after DES implantation. ISR patients are defined as those who had an angiographic minimal lumen diameter (MLD) stenosis ≥ 50% of a stented segment or within 5 mm of a stent edge [1]. Moreover, late lumen loss, reflecting the degree of restenosis, is defined as the difference between poststenting MLD minus MLD at the time of angiographic follow-up. All analyses were performed by two investigators who were blinded to the group information.

### 2.4. Plasma Small sEV Isolation

Venous blood samples were drawn from rats and patients into EDTA-containing vacutainers (BD biosciences, USA). The plasma was obtained by centrifuging at 1600 × g for 20 minutes at 4°C and subsequently stored at -80°C for further experiments. Plasma sEV were purified using differential ultracentrifugation according to the guideline [16]. Briefly, plasma was centrifuged at 10,000 × g for 30 minutes at 4°C to remove cells and debris, then twice at 100,000 × g for 1 hour at 4°C with a SW-41 rotor (Beckman Coulter, USA). The pellets were washed with phosphate buffered saline (PBS) and centrifuged again at 100,000 × g for 1 hour at 4°C to purify the sEV. The isolated plasma sEV were collected and resuspended in 1x PBS for subsequent analysis.

### 2.5. Plasma sEV Identification

After isolation, the morphology of plasma sEV was assessed by transmission electron microscope (TEM, FEI Tecnai G2 spirit). Briefly, 20 *μ*L of sEV suspension was placed on a carbon-coated 200-mesh copper grid for 5 minutes at room temperature and stained with 2% phosphotungstic acid for one minute. Then, the samples were dried for 10 minutes and visualized with TEM at 80 kV. The concentration and size of plasma sEV were analyzed by nanoparticle tracking analysis (NTA) using ZetaView particle tracker (Particle Metrix, Germany). Moreover, protein markers of sEV, such as CD63 (1 : 1000, ab68418, Abcam) and TSG101 (1 : 1000, ab125011, Abcam), were identified by western blots (WB).

### 2.6. Cell Culture

Primary human aortic smooth muscle cells (HASMC) were obtained from American Type Culture Collection (ATCC, PCS-100-012). HASMCs were cultured in Smooth Muscle Cell Growth Basal Medium (ScienCell, 1101) with 2% fetal bovine serum (FBS) at 37°C with 95% humid air and 5% CO_2_. After growing to 70%-80% confluence, cells were washed with PBS and then maintained in Smooth Muscle Cell Growth Basal Medium with 10% exosome-depleted FBS (Gibco, USA) and subsequently incubated with plasma sEV for 24 hours.

### 2.7. sEV Labeling and Uptake

Plasma sEV were labeled with PKH26 Red Fluorescent Cell Linker Kit (Sigma-Aldrich, USA) in accordance with the manufacturer's protocol. Briefly, 100 *μ*L of sEV was added to 150 *μ*L of Diluent C, which were incubated with PKH26 dye (1 *μ*L) Diluent C (250 *μ*L) solution for 4 minutes at room temperature. To terminate the labeling reaction, 500 *μ*L of 1% Bull Serum Albumin (BSA) was added. The labeled sEV were isolated using differential ultracentrifugation as described above to eliminate the excess dye and resuspended in 100 *μ*L of 1x PBS, which were subsequently incubated with HASMC on 24-well plates at 37°C for 6 hours. Then, the images were visualized by confocal microscopy (ZEISS, German).

### 2.8. Concentration of Plasma sEV

BCA Protein Assay Kit (Thermo Scientific, USA) was used to measure the protein concentration in plasma sEV according to the manufacturer's instructions, which has been considered as an index of the number of sEV. The final concentration of plasma sEV was 30 *μ*g/mL in the cell growth medium in vitro, while 20 *μ*g sEV in 100 *μ*L PBS were intravenously injected weekly in vivo.

### 2.9. miRNA Microarray Assay

miRNA microarray was performed by a commercial service (Shanghai OE Biotech Co., Ltd, China). Briefly, total RNAs were extracted from sEV isolated from 2 mL of plasma from ISR patients and control patients. The extracted RNA was labeled and hybridized to an Agilent Human miRNA Microarray Kit (Release 21.0, 8 × 60K), and this microarray contains 2570 probes for mature miRNA. Then, differentially expressed miRNAs between these two groups were screened out using cluster analysis.

### 2.10. Western Blots

Smooth muscle cells and plasma sEV were lysed using RIPA buffer, proteinase inhibitor, and phosphatase inhibitor. Proteins from cultured cells or plasma sEV were quantified with BCA protein assay kits (Beyotime, China). Equal amounts (60 *μ*g) of protein were separated by 10% SDS-PAGE and transferred to PVDF membranes (Millipore, USA), which were then blocked with 5% BSA and incubated overnight at 4°C with individual primary antibodies, followed by incubation with the corresponding secondary antibodies for 2 hours at room temperature. Primary antibodies against CD63 (ab68418), TSG101 (ab125011), *α*-SMA (ab7817), calponin (ab46794), and Samd3 (ab40854) were purchased from Abcam (Cambridge, UK). Primary antibodies against Smad2 (5339), Smad4 (46535), and GAPDH (5174) were acquired from Cell Signaling Technology (Massachusetts, USA). Bands were analyzed by the ImageJ software, and all analyses were performed by two investigators who were blinded to the group information.

### 2.11. Quantitative Real-Time-PCR (qRT-PCR)

Total RNA was extracted using Trizol reagent (Invitrogen) from sEV, HASMC, and carotid artery according to the standard protocol. For sEV-carried miRNA quantification, cel-miR-39 (5 fmol/*μ*L) was added to the isolated RNAs as an exogenous control. For RNA detection in cells and tissues, U6 was set as an endogenous control. The primer sequences for the real-time PCR (RT-PCR) assays were listed in Supplemental Table 1.

### 2.12. Luciferase Reporter Assays

For reporter assays, 293T cells were cotransfected with pmiR-RB-Report™ h-Smad3-WT/-MUT and micrON™ has-miR-501-5p mimic/negative control using Lipofectamine-3000 (Invitrogen) according to the manufacturer's instructions. Firefly and Renilla luciferase activities were analyzed after 48 h using the dual luciferase assay system (Promega, USA) following the manufacturer's instructions.

### 2.13. Cell Transfection of miRNA-501-5p Mimic and Inhibitor

HASMC in 6-well plates were transfected with miR-501-5p mimic (50 nmol/L), miR-501-5p inhibitor (100 nmol/L), or their negative controls (GenePharma, China) using Lipofectamine RNAiMAX (Invitrogen) following the manufacturers' instructions. In the inhibitor experiments, HASMC were transfected with miR-501-5p inhibitor or negative control first, and plasma sEV were added 24 hours later.

### 2.14. miRNA Antagomir Injection

Rats were intravenously injected with antagomir (100 nmol) and negative controls (GenePharma, China) in 200 *μ*L of saline buffer twice a week after the CABI procedure of rats.

### 2.15. Cell Proliferation and Migration Assay

HASMC proliferation was assessed using MTT and EdU assay (Thermo Scientific, USA). Cell migration was measured using Wound Healing and Transwell assay with 8 *μ*m pore size inserts (Corning). Every experiment was repeated three times independently by investigators who did not know the group allocation according to the manufacturers' instructions.

### 2.16. Statistical Analysis

The Shapiro-Wilk normality test was used to assess the distribution of continuous variables. All continuous variables were expressed as mean ± standard error of mean (SEM) and compared using the Student's *t*-test (two groups) or one-way ANOVA followed by Bonferroni's post hoc test (three or more groups). All statistical tests were two-tailed, and a *p* value <0.05 was considered statistically significant. All analyses were performed using the GraphPad Prism 8.0.

## 3. Results

### 3.1. The Association between Plasma sEV and ISR

Study flowchart was summarized in Supplemental Figure 1. sEV were isolated from the plasma of patients with ISR (ISR-sEV) or not (Ctl-sEV) 1 year after coronary stent implantation using differential ultracentrifugation. TEM images showed rounded particles of both ISR-sEV and Ctl-sEV (Figure 1(a)), and NTA revealed a similar size distribution (118.80 ± 1.96 vs. 113.20 ± 1.02 nm) but a higher plasma concentration (9.27 ± 0.15 vs. 5.40 ± 0.06, ×10^11^ particles/mL) of ISR-sEV compared with Ctl-sEV (Figure 1(b)). WB analysis confirmed the presence of sEV marker proteins (Figure 1(c)). We then constructed rat carotid artery stenosis by CABI model, and HE staining showed significant VSMC proliferation 28 days after balloon injury (Figure 1(d)). sEV were purified from the plasma of rats with carotid stenosis (RS-sEV) or sham procedure (Sham-sEV). TEM images revealed rounded particles of both RS-sEV and Sham-sEV (Figure 1(e)), and NTA showed a similar size distribution (134.00 ± 1.21 vs. 133.70 ± 1.92 nm, Supplemental Figure 2(a)) but a higher plasma concentration (3.03 ± 0.03 vs 2.37 ± 0.09, ×10^9^ particles/mL) of RS-sEV than those of Sham-sEV (Figure 1(f)). WB analysis confirmed the presence of sEV marker proteins (Supplemental Figure 2(b)). Taken together, these data showed a relative higher level of plasma sEV in ISR patients and rat carotid artery stenosis.

### 3.2. Plasma sEV Promoting VSMC Phenotypic Modulation

We incubated HASMC with PKH26-labeled plasma sEV, and confocal images found that sEV were internalized by HASMC after a 6-hour incubation (Figure 2(a) and Supplemental Figure 3). Notably, preincubation with ISR-sEV, but not Ctl-sEV, for 24 hours could decrease the expression of HASMC contractile markers *α*-SMA and calponin (Figures 2(b) and 2(c)), and increase HASMC proliferation (Figures 2(d) and 2(e)) and migration (Figures 2(f) and 2(g)). Meanwhile, in vivo study showed the reduced mRNA level of contractile markers (*α*-SMA and calponin) in rat carotid artery stenosis compared with the sham group (Figure 2(h)). In addition, we found that CABI rats treated with RS-sEV could further decrease the expression of *α*-SMA and calponin compared with Sham-sEV treatment (Figure 2(i)). Collectively, these results demonstrated that plasma sEV from ISR patients could promote VSMC phenotypic modulation.

### 3.3. Plasma sEV-Carried miRNA-501-5p and ISR

We performed Agilent human miRNA microarray assay comparing the differential miRNAs between plasma ISR-sEV and Ctl-sEV to explore the possibility of miRNA resulting in ISR-sEV induced VSMC phenotypic modulation. A total of 15 differential miRNAs (fold change ≥ 2.0; *P* < 0.05) of 2570 miRNAs were detected (Figure 3(a)), and 13 upregulated miRNAs of them were further validated by qRT-PCR. qRT-PCR analysis found that miRNA-501-5p was the highest expressed miRNA in plasma ISR-sEV (Figure 3(b)). To further investigate the relationship of plasma sEV-carried miRNA-501-5p and ISR, 20 patients with ISR and 20 patients without ISR 1 year after stent implantation were enrolled, and the baseline clinical characteristics of them are summarized in Supplemental Table 2. Plasma sEV were purified from these 40 patients using differential ultracentrifugation, and we found that sEV-carried miRNA-501-5p level was significantly higher in ISR patients than that in control patients (Figure 3(c)). Furthermore, the level of plasma sEV-carried miRNA-501-5p linearly correlated with late lumen loss (an indicator of the degree of restenosis, *R*^2^ = 0.62, Figure 3(d)). These results suggested that plasma sEV-carried miRNA-501-5p was definitely associated with ISR.

### 3.4. sEV-Carried miRNA-501-5p Promoting VSMC Phenotypic Modulation

To evaluate the functional effects of miRNA-501-5p, transfection with miRNA-501-5p mimic for 24 hours could decrease the expression of HASMC contractile markers *α*-SMA and calponin (Figures 4(a) and 4(b)) and increase HASMC proliferation (Figures 4(c) and 4(d)) and migration (Figures 4(e) and 4(f)). In addition, downregulation of miRNA-501-5p significantly attenuated ISR-sEV-induced HASMC proliferation and migration (Figures 4(g)–4(j) and Supplemental Figure 4-5). To better understand the function of plasma sEV-carried miRNA-501-5p in vivo, we performed qRT-PCR analysis of miRNA-501-5p and its precursor in carotid artery of rats with CABI or RS-sEV treatment. The level of miRNA-501-5p was markedly increased in both CABI rats and RS-sEV-treated rats, but the significant change of pre-miRNA-501-5p level was not found (Figures 5(a) and 5(b)), which indicated that plasma sEV delivered miRNA-501-5p to carotid artery. Furthermore, plasma RS-sEV-treated rats exhibited VSMC proliferation (Figures 5(c) and 5(d) and Supplemental Figure 6) and elevated the media thickness of carotid artery (Figures 5(e) and 5(f)). More importantly, antagomir-501-5p injection could increase the contractile markers *α*-SMA and calponin (Supplemental Figure 7), reverse the VSMC proliferation (Figures 5(c) and 5(d)), and decrease media thickness as well as the ratio of media thickness/lumen diameter in CABI rats by blocking the miRNA-501-5p (Figures 5(e) and 5(f)). Taken together, these results demonstrated that miRNA-501-5p played a crucial role in plasma sEV induced VSMC phenotypic modulation.

### 3.5. Target Gene of miRNA-501-5p in VSMC

By using three online databases, including Targetscan, miRwalk, and miRDB, combining with genes involving in VSMC phenotypic modulation reported by previous articles [17–20], we finally focused on Smad3 as a potential target gene of miRNA-501-5p (Figure 6(a)). GO and KEGG analyses of miRNA-501-5p were also conducted (Supplemental Figure 8-9). Next, luciferase reporter assays were performed with plasmids containing wild-type or mutant Smad3 3′UTR with miRNA-501-5p binding sites (Figure 6(b)). The result showed that miRNA-501-5p could decrease luciferase activity of Smad3 wild-type 3′UTR constructs but had no effect of Smad3 mutated forms (Figure 6(c)). Furthermore, preincubation with miRNA-501-5p mimic markedly inhibited the expression of Smad3 in HASMC (Figure 6(d)). In vivo studies showed decreased mRNA levels of Smad3 in CABI rats (Supplemental Figure 10) and RS-sEV-treated rats (Figure 6(e)) but an elevated level of Smad3 when blocking miRNA-501-5p (Figure 6(f)). Collectively, these results demonstrated that miRNA-501-5p promoted VSMC phenotypic modulation by targeting Smad3.

### 3.6. The Potential Origin of Plasma sEV-Carried miRNA-501-5p

To investigate the potential origins of elevated plasma ISR-sEV-carried miRNA-501-5p, we evaluated the level of miRNA-501-5p and its precursor in the aorta, heart, liver, lung, adipose, and kidney of rats with CABI or not. Both miRNA-501-5p and its precursor markedly elevated only in the aorta and adipose of rats with carotid artery stenosis (Figures 7(a) and 7(b)). Next, the removal of aortic endothelial cells significantly decreased the expression of miRNA-501-5p and its precursor, indicating that endothelial cells might be the major origin of miRNA-501-5p in the aorta (Figure 7(c)). Therefore, we propose that DES implantation increases the production of miRNA-501-5p in multiple tissues, especially in endothelial cells. miRNA-501-5p, cargoed in sEV, is delivered to the VSMC by plasma sEV and promotes VSMC proliferation and migration by targeting Smad3 (Figure 7(d)).

## 4. Discussion

This study for the first-time reports that plasma sEV-carried miRNA-501-5p promotes VSMC phenotypic modulation-mediated ISR through targeting Smad3. There are several major findings in the present study. First, the concentration of plasma sEV in ISR patients was higher compared with non-ISR patients. Second, plasma sEV-carried miRNA-501-5p was identified to enhance VSMC proliferation and migration by targeting Smad3, and the level of plasma sEV-carried miRNA-501-5p linearly correlated with the degree of restenosis. Third, vascular endothelial cells might be the major primary origin of plasma sEV miRNA-501-5p. These findings exhibit a novel mechanism of VSMC-mediated ISR by plasma sEV-carried miRNA-501-5p.

In this study, we investigated the mechanism of VSMC phenotypic modulation-mediated ISR. In the DES era, ISR still remains a therapeutic challenge in spite of the improvements of stent design, novel coating drugs, and polymers. The current opinion [1] is that the underlying mechanisms of ISR are quite complex, at least including mechanical and biologic factors. VSMC is the major cell type in the artery, and fully differentiated/contractile VSMC can maintain the arterial function of contraction/dilation and control normal blood pressure. Differentiated VSMC could switch to a dedifferentiated phenotype to gain the function of proliferation, migration, and ECM synthesis for tissue reparation in response to vessel injury. Imbalanced VSMC switching leads to the excessive VSMC hyperplasia and ECM deposition and ultimately results in artery stenosis. In our study, rats with carotid artery stenosis after balloon injury exhibited decreased expression of contractile markers *α*-SMA and calponin and increased VSMC proliferation compared with rats in the sham group. Our results, in line with previous articles [4, 5, 21], confirmed that VSMC phenotypic modulation plays a crucial role in restenosis.

sEV, small endogenous membrane vesicles released from various cell types, are of great interest because of their extensive participation in cell-to-cell communication [10, 12]. The mean size of most sEV in our study was 110-130 nm, indicating that the sEV are very likely to be exosomes. Several previous studies [4–6, 10, 22] have reported the association of sEV and VSMC phenotypic modulation at the level of cell and animal experiment, but evidence from patient level still remains insufficient. In our study, we purified plasma sEV directly from ISR patients and found that the concentration of plasma sEV in ISR patients was higher than that in non-ISR patients. More importantly, these plasma sEV could be internalized by VSMC and decrease the expression of VSMC contractile markers *α*-SMA and calponin and increase VSMC proliferation and migration.

sEV harbor proteins, miRNAs, and mRNAs and deliver these signals to receptor cells through systemic circulation. In fact, miRNAs, as a class of epigenetic factors, have been reported to drive VSMC toward the differentiated/contractile phenotype, including miRNA 1 [23], miRNA-124 [24], miRNA-143/145 [6], and miRNA-663 [25]. In response of vascular injury, several miRNAs, such as miRNA-206 [26], miRNA-221 [9], and miRNA-222 [27], could switch VSMC toward the dedifferentiated/synthetic phenotype to tissue reparation. With new-generation sequencing and qRT-PCR validation in plasma sEV from patients, we found that miRNA-501-5p was markedly elevated in ISR patients or CABI rats. miRNA-501-5p is a relative novel miRNA and has been reported to promote cell proliferation and migration in the development of cancer [28–30]. Similarly, in our study, plasma sEV-carried miRNA-501-5p decreased the expression of VSMC contractile markers *α*-SMA and calponin, increased VSMC proliferation and migration, and exhibited profound function of promoting VSMC phenotypic modulation both in vivo and in vitro. More importantly, the level of plasma sEV-carried miRNA-501-5p linearly correlated with the degree of restenosis, which provides a possibility for potential clinical application.

Further bioinformatic analysis and validation experiments showed that Smad3 is target of miRNA-501-5p in VSMC. It is well established that Smad3 plays a crucial role in maintaining the differentiated/contractile phenotype of VSMC [17, 20], and loss of Smad3 can increase VSMC proliferation and reduce expression of VSMC contractile markers [18, 19]. Consistent with these studies, our data found that miRNA-501-5p markedly reduced the expression of *α*-SMA and calponin and promoted VSMC proliferation and migration in vitro by inhibiting Smad3 expression. Meanwhile, in vivo study with suppressing miRNA-501-5p showed the increased expression of Smad3 and VSMC contractile markers and the decreased VSMC proliferation in carotid artery.

Furthermore, we investigated the potential origins of increased plasma sEV-carried miRNA-501-5p. We found that both miRNA-501-5p and its precursor pre-miRNA-501-5p significantly elevated in the aorta and adipose. Notably, the removal of aortic endothelium could markedly reduce the expression of miRNA-501-5p and its precursor, elucidating that endothelial cells might be the major origin of miRNA-501-5p. Our data, in line with previous study [31], indicated that endothelial cells are the important origin of plasma sEV-carried miRNAs.

There are several limitations in the present study. First, we found plasma sEV-carried miRNA-501-5p promoted VSMC phenotypic modulation-mediated ISR by targeting Smad3, but we could not rule out a possibility of other miRNAs and other targets of miRNA-501-5p. Second, although CABI rat is a widely used in vivo model for studying VSMC phenotype, this model cannot simulate the situation of ISR after stent implantation completely. Third, our study found endothelial cells might be the major origins of the increased plasma sEV-carried miRNAs, but other tissues could not be totally excluded because of the lack of further validation.

## 5. Conclusion

Plasma sEV in ISR patients are elevated and play a crucial role in VSMC phenotypic modulation. miRNA-501-5p was identified in plasma sEV to enhance VSMC proliferation and migration by targeting Smad3. Vascular endothelial cells might be the major origin of plasma sEV miRNA-501-5p. Collectively, these findings showed that plasma sEV-carried miRNA-501-5p promotes VSMC phenotypic modulation-mediated ISR through targeting Smad3.

## Figures and Tables

**Figure 1:** Characterization and function of plasma sEV from patients and rats. The isolated small extracellular vesicles (sEV) from patients with in-stent restenosis (ISR) or not (control) were used for the characterization. (a) Representative transmission electron microscopic (TEM) images of sEV. (b) Representative results of nanoparticle tracking analysis (NTA) demonstrating the particle distribution of sEV (*n* = 3). (c) Representative western blots identifying the biomarkers of sEV including CD63 and TSG101 in the same amount of plasma sEV. (d) Representative hematoxylin-eosin stained images of carotid arteries from rat carotid artery balloon injury (CABI) model or sham group (*n* = 6). (e) Representative TEM images of sEV from rats. (f) NTA showing the concentration of sEV (*n* = 3). Values are mean ± SEM. ^∗∗^*P* < 0.01 and ^∗∗∗^*P* < 0.001. Ctl-sEV: sEV purified from the plasma of patients without ISR after stent implantation; ISR-sEV: sEV purified from the plasma of patients with ISR after stent implantation; Sham-sEV: sEV purified from the plasma of rats with sham procedure; CABI-sEV: sEV purified from the plasma of rats with carrotid artery stenosis after balloon injury.

**Figure 2:** The effect of plasma sEV from patients on vascular smooth muscle cells proliferation and migration. (a) Primary human aortic smooth muscle cells (HASMC) were cultured in the presence of PKH26-labeled sEV. Representative confocal images showing the red sEV and the blue nuclei (DAPI) of HASMC. (b) Representative blots and quantified data showing the expression of vascular smooth muscle cell- (VSMC-) specific contractile marker (*α*-SMA and calponin) in HASMC treated with plasma sEV. (c) Representative confocal images showing immunofluorescent staining for VSMC-specific contractile marker (*α*-SMA, green) to determine VSMC identity. Nuclei were stained with DAPI (blue). The VSMC proliferation was evaluated with Edu-positive cells (d) and MTT assay (e) in HASMC treated with plasma sEV. The VSMC migration was measured using Transwell (f) and wound healing assay (g) in HASMC treated with plasma sEV. (h) The reduced mRNA expression of VSMC-specific contractile markers (*α*-SMA and calponin) in CABI group (*n* = 6). Data are normalized to U6. (i) The further reduced mRNA expression of VSMC-specific contractile marker (*α*-SMA and calponin) in CABI rats treated with sEV (*n* = 6). Values are mean ± SEM. ^∗∗^*P* < 0.01 and ^∗∗∗^*P* < 0.001.

**Figure 3:** miRNA microarray assay and the relationship of miRNA-501-5p and in-stent restenosis. (a) miRNA microarray assays were performed in plasma sEV purified from patients with in-stent restenosis (ISR) or not (*n* = 3). (b) qRT-PCR analysis of the 13 upregulated miRNAs in ISR-sEV and Ctl-sEV (*n* = 3). Data are normalized to cel-miRNA-39. (c) qRT-PCR analysis of plasma sEV-carried miRNA-501-5p level in patients with ISR or not (*n* = 20). Data are normalized to cel-miRNA-39. (d) The relationship between plasma sEV-carried miRNA-501-5p level and late lumen loss (reflecting the degree of restenosis) (*n* = 20). Data are normalized to cel-miRNA-39. ^∗^*P* < 0.05 and ^∗∗^*P* < 0.01.

**Figure 4:** The effect of miRNA-501-5p on smooth muscle cell proliferation and migration. (a) Representative blots and quantified data showing the expression of vascular smooth muscle cell- (VSMC-) specific contractile marker (*α*-SMA and calponin) in primary human aortic smooth muscle cells (HASMC) transfected with miRNA-501-5p mimic. (b) Representative confocal images showing immunofluorescent staining for VSMC-specific contractile marker (*α*-SMA, green) to determine VSMC identity. Nuclei were stained with DAPI (blue). The VSMC proliferation was evaluated with Edu-positive cells (c) and MTT assay (d) in HASMC transfected with miRNA-501-5p mimic. The VSMC migration was measured using Transwell (e) and wound healing assay (f) in HASMC transfected with miRNA-501-5p mimic. Effects of miRNA-501-5p inhibitor on MTT assay (g), immunofluorescent staining of *α*-SMA (h), Edu assay (i), and transwell assay (j), in HASMC treated with plasma sEV, then transfected with miRNA-501-5p inhibitor or not. *n* = 8 per group in (d) and (g); *n* = 3 per group in other groups. NC: negative control. Values are mean ± SEM. ^∗^*P* < 0.05, ^∗∗^*P* < 0.01, and ^∗∗∗^*P* < 0.001.

**Figure 5:** Plasma sEV-carried miRNA-501-5p promotes rat carotid artery stenosis. (a) qRT-PCR analysis of pre-miRNA-501-5p and miRNA-501-5p in carotid artery from rats with carotid artery balloon injury (CABI) or sham procedure. Data are normalized to U6. (b) qRT-PCR analysis of pre-miRNA-501-5p and miRNA-501-5p in carotid artery from CABI rats treated with plasma sEV. Data are normalized to U6. (c) Representative hematoxylin-eosin stained images of carotid arteries from CABI rats treated with plasma sEV or antagomir-501-5p. (d) Representative Masson stained images of carotid arteries from CABI rats treated with plasma sEV or antagomir-501-5p. (e and f) Quantitative analysis for media thickness and the ratio of media thickness and lumen diameter. *n* = 6 for each group. Values are mean ± SEM. ^∗∗^*P* < 0.01 and ^∗∗∗^*P* < 0.001.

**Figure 6:** Smad3 is target gene of plasma sEV-carried miRNA-501-5p in smooth muscle cells. (a) Screening scheme for putative target gene of miRNA-501-5p. (b) Schematic of miRNA-501-5p putative target sites in the 3′URT of Smad3 and the sequences of mutant UTRs. (c) Dual luciferase reporter assay of 293T cells cotransfected with miRNA-501-5p mimic or negative control (NC) (*n* = 3). (d) Representative blots and quantified data showing protein expressions of Smad2, Smad3, and Smad4 in human aortic smooth muscle cells (HASMC) transfected with miRNA-501-5p mimic or NC (*n* = 3). (e) qRT-PCR analysis of Smad2, Smad3, and Smad4 in carotid artery from rats with carotid artery balloon injury (CABI) undergoing sEV injection (*n* = 6). Data are normalized to U6. (f) qRT-PCR analysis of Smad2, Smad3, and Smad4 in carotid artery from rats with carotid artery balloon injury (CABI) undergoing antagomir-501-5p injection (*n* = 6). Data are normalized to U6. Values are mean ± SEM. ^∗∗^*P* < 0.01 and ^∗∗∗^*P* < 0.001.

**Figure 7:** The potential origin of miRNA-501-5p and the proposed schematic. qRT-PCR analysis of miRNA-501-5p (a) and pre-miRNA-501-5p (b) in tissues from rats with carotid artery balloon injury (CABI) or not. Data are normalized to U6 (*n* = 6). (c) qRT-PCR analysis showing that the expressions of miRNA-501-5p and pre-miRNA-501-5p are significantly higher in rat aorta with endothelium (endo+) than that without endothelium (endo-). Data are normalized to U6 (*n* = 6). (d) Drug-eluting stent implantation increases the production of miRNA-501-5p in multiple tissues, especially in endothelial cells. miRNA-501-5p, cargoed in sEV, is delivered to the vascular smooth muscle cells (VSMC) by plasma sEV and promotes VSMC proliferation and migration by targeting Smad3. Values are mean ± SEM. ^∗^*P* < 0.05, ^∗∗^*P* < 0.01, and ^∗∗∗^*P* < 0.001.

## Data Availability

The data used to support the results of this study are included within the article.

## Supplementary Materials

Supplementary Materials Supplemental Figure 1: study flowchart. Supplemental Table 1: the primer sequences for RT-PCR assays. Supplemental Table 2: clinical characteristics of enrolled patients. Supplemental Figure 2: identification of plasma small extracellular vesicles (sEV). Supplemental Figure 3: PKH26-labeled sEV internalized by human aortic smooth muscle cells (HASMC). Supplemental Figure 4: miRNA-501-5p inhibition and vascular smooth muscle cells (VSMC) contractile markers. Supplemental Figure 5: miRNA-501-5p inhibition suppressing VSMC migration. Supplemental Figure 6: plasma sEV-carried miRNA-501-5p and VSMC proliferation. Supplemental Figure 7: miRNA-501-5p inhibition and VSMC contractile markers of rats. Supplemental Figure 8: GO analyses of miRNA-501-5p. Supplemental Figure 9: KEGG analysis of miRNA-501-5p. Supplemental Figure 10: *α*-SMA and Smad3 expression in carotid artery of rats.
